The article "Feasibility Analysis and Countermeasures of Psychological Health Training Methods for Volleyball Players Based on Artificial Intelligence Technology" was published in 2022. Journal: J Environ Public Health.

# Feasibility Analysis and Countermeasures of Psychological Health Training Methods for Volleyball Players Based on Artificial Intelligence Technology

**DOI:** 10.1155/2022/6486707

**Published:** 2022-08-25

**Authors:** Xiaoyu Jin

**Affiliations:** Institute of Physical Education, Ludong University, Yantai, Shandong 264025, China

## Abstract

In the process of volleyball players' mental health training, there exists the problem of low parameter accuracy. In order to further improve the accuracy of mental health training methods, based on artificial intelligence calculation, the neural network and long and short-term memory network were used to analyze the model. Estimation algorithm was used to describe the data, and finally, the optimization model was obtained to describe the feasibility study of mental health. In addition, the relevant data were used to verify and analyze the model. The research shows that in the time update curve, with the increase of the model state, the corresponding curve on the whole first presents a fluctuating trend of different degrees. The increase of model state will make the corresponding time value gradually tend to flat. The fluctuation of the corresponding time index is obvious. Indicators corresponding to the status update curve show an obvious linear change trend with the increase in time, and the overall linear characteristics are obvious. This shows that when time is constant, the relationship between the corresponding parameter and the state value conforms to the linear law. The corresponding state index gradually increases and eventually tends to be stable. Through the analysis, it can be seen that the proportion of different indicators under the effect of artificial intelligence and the calculation results are different. The parameters show an obvious linear variation trend, indicating that the corresponding model parameters can well reflect the data changes. Finally, the accuracy of the model is verified by the method of experimental comparison. The relevant research results can provide a new model and a method for volleyball players' mental health training.

## 1. Introduction

Artificial intelligence technology plays different roles in different fields: digital device technology [1], College English education [2], medical surgery [3], and industrial manufacturing [4]. In the field of industrial design, conversion system plays an important role. Conversion system can improve the speed and efficiency of industrial design through calculation and analysis. However, the existing industrial conversion system has the problem of high energy consumption, which will further restrict the development of industrial conversion. In order to further improve the efficiency and speed of industrial conversion, artificial intelligence calculation was used to estimate the original conversion system. Neural network and long and short-term memory models were used to improve the calculation accuracy of data [5], so as to obtain the optimized model data. And a new computing model was used to further optimize the data, so as to obtain an accurate, high school, clean conversion system. Finally, data was used to verify the accuracy of the model. With the development of science and technology, intelligent English teaching has made continuous progress, but there were still some problems such as chaos in teaching class. Based on the theory of artificial intelligence, neural network algorithm was used to extract the classroom indicators, and an optimized intelligent classroom computing model was obtained through analysis [6]. Through this model, the classroom can be dynamically adjusted, thus greatly improving the efficiency of English teaching. Finally, relevant cases can be used to verify the accuracy of the model and predict the intelligent teaching of some classes.

The above studies were mainly aimed at classroom education and industrial design and other fields. There were relatively few researches on psychological health training methods for volleyball players. And volleyball players' mental health education and training for improving athletes' sports skills was very important. Based on artificial intelligence technology, this study adopts neural network, long and short-term memory model, and Kalman filter algorithm to analyze the original data. Besides, the estimation calculation method was used to further extract the data, so as to obtain the feasibility model describing the mental health training method. The model can analyze the data under different indexes and find out the optimal calculation results. Finally, the optimization model was verified by comparing the data with the model. This research can provide support for the application and analysis of artificial intelligence technology in other fields, and provide a reference for the training methods of volleyball players.

## 2. Estimation Algorithm of Artificial Intelligence Model

As a sub-discipline of computer science, artificial intelligence is the study of computational models of intelligent behavior and the development of computational systems with thinking activities such as perception, reasoning, learning, association, and decision making [7, 8]. Artificial intelligence solves complex problems that require human intelligence. In short, artificial intelligence is represented and performed by computers. In recent years, the research field of artificial intelligence is expanding, including automatic planning, expert system, production system, and so on [9, 10]. The advantages of artificial intelligence technology mainly include the following aspects: (1) Advanced infrastructure: Artificial intelligence technology, especially machine learning and deep learning applications, can perform best on servers with multiple high-speed graphics processing units running in parallel. (2) Low cost: Artificial intelligence technology not only eliminates the need to pay for expensive hardware but also allows organizations to pay only for the hardware they use. (3) Scalability: As with other types of cloud services, artificial intelligence technology makes it very easy to scale.

Theories related to artificial intelligence technology are widely used in volleyball and other fields. In order to further analyze the calculation process of artificial intelligence technology, the calculation flow chart of artificial intelligence technology is drawn as shown in Figure 1. It can be seen from the figure that volleyball-related data should be imported into the flow chart first, and then initialization quantum population algorithm is adopted to analyze initialization parameters. Then, the corresponding parameter algorithm will be set, and the parameters will be further iterated through the parameter algorithm, and further analysis will be carried out through the quantum observation operation, quantum evolution operation, and quantum evaluation operation. So that the corresponding optimization parameters can meet the requirements of the model. In order to judge whether the parameters meet the requirements of the model, it is necessary to judge the termination conditions. If it meets the requirements, the feasibility calculation results of the optimal technical parameters shall be output; if it does not meet the requirements, it shall be imported into the quantum update operation module. Through the iterative operation of quantum update, the corresponding data is imported into the quantum observation operation data for iterative analysis until the requirements are met.

### 2.1. Kalman Filtering Algorithm

Artificial intelligence technology can be divided into three main computing methods [11, 12]: Kalman filter algorithm, neural network algorithm, and long and short-term memory algorithm according to the different research content [13, 14]. Kalman filter is a linear system state equation, through the system input and output observation data, the optimal estimation of system state algorithm.

The classical Kalman filter algorithm is mainly aimed at linear system, while the classical Kalman filter algorithm cannot be used directly for the non-linear system of volleyball players' mental health training, so the extended Kalman filter algorithm needs to be used [15, 16]. Based on classical Kalman filter, the extended Kalman filter transforms the non-linear state space equation of the system into a linear state space equation by using first-order Taylor expansion. The standard Kalman filter equation is mainly composed of time update module and state update module, and its specific equation is shown as follows:.

(1) Time update. The time quantity corresponding to the time state is a random quantity, so it is impossible to measure the exact value, but it can be estimated according to some statistical point of view according to a series of observations. An optimal estimate approximates the true value as accurately as possible. The time state quantity can be analyzed by using optimal estimation. The corresponding time update algorithm formula is as follows:
  (1) $$\begin{array}{c} X_{k}=A_{k-1}\times X_{k-1}+B_{k-1}\times U_{k-1}, \end{array}$$
  (2) $$\begin{array}{c} P_{k}=A_{k-1}\times p_{k-1}+A_{k-1}^{T}\times Q_{k-1}. \end{array}$$
In order to further study the influence of different parameters in the Kalman filter algorithm in artificial intelligence on the calculation results, the corresponding time update formula is obtained through calculation. The time update formula can be used to analyze different model parameters, and it can be seen from the analysis that different formulas can better reflect the change degree of time update. In order to quantitatively describe such updating degree, time updating curves under the action of four different parameters are drawn through analysis, as shown in Figure 2. It can be seen from Figure 2 that four different curves have different manifestations under different calculation states: As can be seen from the curve corresponding to parameter *A*, with the gradual increase of the state, the corresponding time quantity shows *A* trend of slow increase first, then gradual decline and then fluctuation. When its iteration state exceeds 225, the curve gradually tends to be flat. It can be seen from the curve corresponding to parameter *X* that it also shows a trend of increasing first and then decreasing, but its fluctuation range is relatively large. The curve still shows a gradual change trend. As can be seen from the curve corresponding to parameter *B*, with the gradual increase of iteration state, the corresponding time value gradually decreases. The downward slope of the curve is approximately constant, and then when the iteration state exceeds about 150, the curve gradually tends to be flat. According to the change of the curve corresponding to parameter *U*, it can be seen that with the gradual increase of iteration state, the corresponding curve drops slowly at first, and then gradually tends to flat when the curve reaches the highest point. According to the curves corresponding to the four different states, it can be seen that the curve corresponding to parameter *A* has the greatest change, while the change of curve *U* is relatively small, while the change of curve *A* and curve *B* is basically the same. Finally, the corresponding time state curve is obtained. From the change of time state curve, it can be seen that its change range can better reflect the change trend of different parameters. First, the curve gradually increases rapidly and then decreases slowly. Finally, it gradually tends to a gentle overall change trend. It should be noted that the four parameters can update the corresponding data changes in a better response time.
(2) Status update: state estimation is an important part of the Kalman filter. Generally speaking, it is an estimation problem to make quantitative inference of random quantity according to the observation data, especially for the state estimation of dynamic behavior, which can realize the estimation and prediction function of a real-time running state. The corresponding algorithm formula is as follows:
  (3) $$\begin{array}{c} \left\{\begin{array}{c} K_{k}=P_{k-1}\times H_{k-1}^{T}\times {\left[H_{k-1}\times P_{k-2}\times H_{k-1}^{T}+R_{k-1}\right]}^{-1},\\ X_{k}=X_{k-1}\times K_{k-1}\times \left[Z_{k-1}-H_{k-1}\times X_{k-1}\right],\\ P_{k}=\left[I-H_{k-1}\times K_{k-1}\right]\times P_{k-1}. \end{array}\right. \end{array}$$

Through the above analysis, it can be seen that the time change curve in different states has different trends, and the analysis shows that the time update can also have a certain influence on the state. Therefore, in order to better analyze the change rule of state update, several different state change curves are drawn, as shown in Figure 3. It can be seen from Figure 3 that the curves under the action of four different parameters have different variation trends. According to the change curve corresponding to parameter *K*, it can be seen that the curve drops rapidly at first, then gradually decreases to the lowest point and tends to be constant. In the previous stage, the curve presents an obvious linear downward trend. According to the curve corresponding to parameter *H*, it can be seen that the curve has an obvious linear increasing trend, and the overall trend is gradually increasing. This indicates that the parameter has a good linear correlation with the status data. The curve corresponding to parameter *P* also has a good linear correlation, and its corresponding slope is higher than the curve corresponding to parameter *H*. It can be seen from the curve corresponding to parameter I that with the gradual increase of time, the corresponding curve shows obvious fluctuation phenomenon, but the fluctuation range is relatively small, and the overall approximately constant at about 38. Through the above calculation and analysis, the corresponding state value is finally obtained. With the gradual increase of time, the corresponding state curve increases slowly at first and then gradually tends to be stable, with a relatively large range of change, which can better reflect the change rule of time.

### 2.2. Neural Network Algorithm

Artificial neural network, or short-form neural network, is a mathematical model that simulates the structural operation characteristics of animal neural network [17, 18]. Neural network algorithm is an adaptive non-linear dynamic system composed of a large number of simple basic components. The structure and function of each neuron are relatively simple, but the system behavior produced by the combination of a large number of neurons is very complex. It can process information by adjusting the weight ratio and threshold value connected between a large number of internal nodes. More and more researchers have applied their outstanding performance abilities such as strong non-linear fitting ability and good generalization to the feasibility estimation of mental health training [19, 20].

In order to further analyze the calculation process of neural network algorithm and better study, the calculation of artificial intelligence technology, the neural network calculation process and corresponding learning method are obtained through analysis and summary, as shown in Figure 4. It can be seen from the computation flow of neural network that the model has an obvious input layer, hidden layer, and output layer, which belongs to the characteristic of neural network computation. Firstly, the corresponding data will be imported to the input layer, and the redundant data will be eliminated through the input layer, and the corresponding data will be imported to the hidden layer, and the optimized data will be obtained through the calculation of the hidden layer. Then, the optimized data can be imported into the output layer for further output calculation, and the corresponding optimized data can be imported into the model for further analysis through the corresponding learning method, so as to output the data. It can be seen from the corresponding learning method that the input data is first input into the neural network for calculation, and then imported into the comparison module for comparison with the original target value. Through comparison, it can be seen that if the data meets the requirements, the data will be output; if not, the corresponding weights will be adjusted, and then it will be imported into the neural network again for iterative calculation until the requirements are met.

Neural network is one of the most widely used neural networks at present [21, 22]. It is a network structure model of forward solution and backpropagation. The typical neural network consists of input layer, hidden layer, and output layer. The network is composed of multiple neurons as a unit. The relationship between each parameter is shown in the following formula:

(4) $$\begin{array}{c} O=f\times \left[\sum_{i}^{n}W_{ij}x_{i}-T_{j}\right], \end{array}$$

where *x*_i_ is the input of the neuron, *w*_*ij*_ is the input weight of the neuron, *T*_*j*_ is the threshold, *f* represents an activation function, and *O* represents the output of the neuron.

The parameters under the action of neural network have a certain change relationship, and the analysis shows that the change relationship is typical non-linear change. Therefore, the change rule of different parameters can be analyzed, so as to better grasp the change rule of neural network. According to the different properties of parameters, parameters can be divided into three main parts: weight, function, and threshold. Therefore, the variation relationship among the corresponding three parameters is obtained through calculation, and the corresponding curve is shown in Figure 5. It can be seen from the weight curve that with the gradual increase of the input value, the corresponding output value increases slowly at first and then presents a linear downward trend. When the data corresponding to the curve drops to the lowest point, the curve gradually increases with the further increase of the value, and then presents a relatively gentle change. The overall non-linear characteristics are relatively obvious. It can be seen from the corresponding function curve that the initial value still shows an increasing trend. With the further increase of input data, the curve drops rapidly to the lowest point and then gradually tends to be gentle. Although the curve still fluctuates to a certain extent in the process of increasing input data, the overall variation range of output value is relatively small. As can be seen from the corresponding threshold curve, with the increase of the corresponding input value, the curve drops rapidly at first, and then shows a trend of rapid decline. The overall volatility is relatively obvious and the range of variation is relatively large, so its influence on the model is the greatest.

It can be seen from the analysis that the activation function of neurons has a great influence on the calculation and change of input and output characteristics of neurons. According to different needs, there are many types of activation functions, including threshold function, non-linear function, piecewise linear function, and probability function. The classic activation function is the Sigmoid function, whose output expression is:

(5) $$\begin{array}{c} f\left(x\right)=\text{sigmoid}\left(x\right)=\frac{1}{1+e^{-x}}. \end{array}$$

It can be seen from the above formula that different types of activation functions have different manifestations. By changing the *x* value of the activation function, the corresponding experimental value and the *y* change data of the calculated value were obtained, and then the corresponding activation number change was obtained, as shown in Figure 6. It can be seen from Figure 6 that curves under the action of test values have obvious linear characteristics. In the process of gradual increase of independent variable *x*, the *y* value corresponding to the curve also shows a trend of rapid increase, and the corresponding *y* value is relatively small when it increases to the highest point. From the change curve of the calculated value of the activation function, it can be seen that with the gradual increase of the independent variable *x*, the corresponding *y* also shows an obvious linear change trend. When it reaches the highest point, the corresponding *y* is relatively large. Through the changes in the two curves, it can be seen that the slope of the calculated value of the activation function is greater than that of the corresponding experimental value. Therefore, when selecting the specific function value, the corresponding analysis of the test data should be carried out, so that the corresponding results can meet the calculation needs of the test value. At the same time, the activation function corresponding to the test value can be optimized and analyzed to reduce its corresponding change value, so as to better conform to the change rule of the test value.

### 2.3. Long and Short-Term Memory Networks and Evaluation

Long and short-term memory network can solve the problem of memory forgetting over long distances [23, 24]. The main difference lies in that the processing of information in neural network becomes more precise. The long and short-term memory network has three gates to protect and control the cellular state, including the forgetting gate, input gate, and output gate [25, 26]. Long and short-term memory network has similar control flow to the basic recursive neural network, but the control logic inside the basic unit of long and short-term memory network is slightly more complex. The core component of the long-term memory network is the basic unit, which contains several control structures to process data in a sequence. The gating structure of long and short-term memory network solves the short-term dependence problem effectively. Long and short-term memory network model is good at modeling the whole time continuous sequence and capturing the long-distance dependence information. Long and short-term memory network is a temporal recursive neural network that is suitable for processing and predicting important events with relatively long intervals and delays in time series. Long and short-term memory network is a special kind of recurrent neural network which is proposed to solve the error problem in the structure. The output gate filters the information to be output to the next time step and selectively retains and removes some previous data. The corresponding network calculation formula is as follows:

(6) $$\begin{array}{c} O_{t}=\sigma \times \left[W_{0}\times \left(h_{t-1},x_{t}\right)+b_{0}\right], \end{array}$$

(7) $$\begin{array}{c} h_{t}=o_{t}\times \;\tan\;h\left(C_{t}\right), \end{array}$$

where *σ* is the number of layers; *h* is the output network.

In order to better analyze the calculation process of long and short-term memory network, the output results under the action of different layers and corresponding output grids were obtained through analysis and calculation. The corresponding result is shown in Figure 7. As can be seen from the output results, the corresponding input results increase slowly at first with the increase of the number of layers, and when it reaches the local highest point, the curve decreases slowly with the increase of the number of layers. With the further increase in the number of layers, the curve still shows an obvious increasing trend, and its increasing slope is higher than that of the first stage, indicating that the change range of this stage is relatively large. When the number of corresponding layers increases again, the output of the curve shows a slow downward trend, and the overall fluctuation of the curve is obvious. It can be described by the method of non-linear characteristics, and its non-linear characteristics can reflect the complexity and practicability of long and short-term memory network.

In order to better analyze the calculation results of different network calculation methods, different indicators are used to estimate the model [27, 28]. The corresponding evaluation indicators of the estimation model algorithm are as follows:

(1) Mean absolute error: mean absolute error is also called mean absolute deviation, and its formula is as follows:
  (8) $$\begin{array}{c} \text{MAE}=\frac{1}{n}\sum_{i=1}^{n}\left|x_{i}-y_{i}\right|. \end{array}$$
(2) Mean square error: mean square error is a measure reflecting the difference between the estimated quantity and the estimated quantity, and its formula is as follows:
  (9) $$\begin{array}{c} \text{MSE}=\frac{1}{n}\sum_{i=1}^{n}{\left(x_{i}-y_{i}\right)}^{2}. \end{array}$$
(3) Root mean square error: root mean square error is consistent with mean square error in substance, and its formula is as follows:
  (10) $$\begin{array}{c} \text{RMSE}=\sqrt{\frac{1}{n}\sum_{i=1}^{n}{\left(x_{i}-y_{i}\right)}^{2}}. \end{array}$$
(4) R squared: *R* squared is the ratio of the sum of the squares of regression and the sum of the squares of total deviation, and its formula is as follows:
  (11) $$\begin{array}{c} R^{2}=1-\frac{\left(\sum_{i}{\left(x_{i}-y_{i}\right)}^{2}/n\right)}{\sum_{i}{\left(x_{i}-\bar{y}\right)}^{2}/n}, \end{array}$$
  where $\bar{y}$ represents an expectation of the sequence of target values.

It can be seen from the above calculation formula that the results obtained by the evaluation method of the estimation model have different trends. In order to better analyze the change curves corresponding to the four different error evaluation methods, the evaluation curves are obtained by summarizing, analyzing, and calculating, as shown in Figure 8. It can be seen from Figure 8 that the curve of mean absolute error increases slowly at first and then tends to be flat with the gradual increase of samples. With the increase of corresponding sample samples again, the curve gradually tends to be stable. After the stability, the curve rapidly increases to the maximum value when the corresponding time reaches about 80, and then gradually tends to be stable. It shows that the error corresponding to this index has typical linear and non-linear characteristics and can well reflect the calculation results of long and short-term memory network. As can be seen from the change curve of mean square error, it presents a typical two-stage linear change characteristic. First of all, with the gradual increase of samples, the corresponding curves decline slowly first, and the corresponding curves decline amounts are basically the same, indicating that their linear characteristics are relatively obvious. When the sample reaches about 85, the curve increases rapidly to a local peak, and then gradually tends to be stable. The reason for the rapid increase of the curve is that the corresponding data has certain volatility in the calculation process. It can be seen from the change curve of root mean square error that it increases slowly at first and then decreases gradually, showing local inverted U-shaped change. With the increase of samples, the curve increases rapidly to the maximum value, which indicates that the curve can well show an obvious linear change relationship with the corresponding error. It can be seen from the *r*-squared curve that the curve increases slowly first, then decreases slowly, and then increases rapidly to the maximum value. With the gradual increase of samples, the corresponding curve shows the change law of linear decline. Several different error indicators can better reflect the change law of different data. The corresponding data change curve increases linearly to the highest value at first, and slowly decreases to the lowest point with the gradual increase of samples, and finally tends to be stable. In the selection process of several different indicators, the change characteristics of indicators should be considered comprehensively, so as to better reflect the law of data change.

## 3. Research on Estimation Algorithm Based on Artificial Intelligence Calculation

The estimation methods based on artificial intelligence can be divided into two different types according to different calculation principles: the estimation model of neural network algorithm and the estimation model of long and short-term memory network algorithm [29, 30].

### 3.1. Estimation Model of Neural Network Algorithm

Neural network can arbitrarily fit the relationship between input and output, and there is no corresponding system error that leads to a large estimation error [31, 32]. The estimation accuracy of neural network in mental health training is relatively high, and its network model size can be balanced and adjusted with the estimation accuracy, so as to control its model size for subsequent deployment and application in embedded systems. Since the input data of the selected neural network are different types of data, inconsistent units of measurement are easy to make the neural network difficult to converge and lead to large errors. For the neural network algorithm itself, the important factor affecting the estimation result is the selection of input and output parameters. For the selection of input layer variables, it is necessary to consider that variables have a certain impact on the model itself. A reasonable selection of input features is conducive to improving the accuracy of model estimation. In addition, it is also necessary to consider the difficulty of measuring input variables. Therefore, it is necessary to normalize the data and fix the input data within a certain range. The commonly used normalization formula is as follows:

(12) $$\begin{array}{c} \bar{x}=\frac{x_{i}-x_{\min}}{x_{\max}-x_{\min}}, \end{array}$$

where $\bar{x}$ represents the normalized data; *x*_i_ stands for raw data; *x*_min_ and *x*_max_ represent the maximum and minimum values of the same variable, respectively. The quality of the initial weight of the network will directly affect the length of the network training, and the initial weight is generally set as a random number between −1 and 1, rather than a direct value of 0.

The number of hidden layer nodes also has a great influence on the performance of the whole neural network. In general, multiple networks with different numbers of hidden layer nodes can be tested to test the generalization error of each network and select an optimal network with the corresponding number of hidden layer nodes. If the hidden layer nodes are too low or too high, the accuracy of the model will be affected. Therefore, an appropriate number of hidden layer nodes should be selected to ensure a small generalization error of the whole.

In order to better describe the estimation model under the action of neural network, the conventional method is used to analyze the normalization formula, and the corresponding relationship between the normalized data and the maximum and minimum values can be obtained through the analysis. In order to better explain the change rules of maximum and minimum values and normalized data, the corresponding normalized curves are drawn, as shown in Figure 9. As can be seen from the curve, with the gradual increase of distance, the corresponding minimum value is relatively stable. And the corresponding value is relatively small, but with the gradual increase of sample distance, the curve increases rapidly to the local maximum value, and a certain jump phenomenon occurs. With the further increase in sample distance, the curve shows a gradually increasing trend. It can be seen from the change curve of the maximum value that the data first slowly drops to the lowest point, and then gradually increases with the distance. It can be seen from the analysis that the non-linear characteristics of the normalized data corresponding to the maximum value are more obvious than that of the minimum value, which can better reflect the change rule of the planning data.

### 3.2. Estimation Model Based on Long- and Short-Term Memory Network Algorithm

Compared with neural network algorithm, network model with long and short-term memory ability is more suitable for calculating the feasibility data of volleyball players' mental health training [33, 34]. Therefore, its accuracy is better than that of neural network in the estimation of training methods. There are several common model loss functions to solve regression problems, and the loss functions of the three are shown as follows.

(a) Squared loss function
  (13) $$\begin{array}{c} Y={\left(y-f\left(x\right)\right)}^{2}. \end{array}$$
(b) Absolute value loss function
  (14) $$\begin{array}{c} Y=\left|y-f\left(x\right)\right|. \end{array}$$
(c) Classification loss function
  (15) $$\begin{array}{c} Y=\left\{\begin{array}{cc} \frac{1}{2}{\left(y-f\left(x\right)\right)}^{2} & \left|y-f\left(x\right)\right|\leq \delta ,\\ \delta \left|y-f\text{(}x\text{)}\right|-\frac{1}{2}\delta^{2} & \left|\left.y-f\text{(}x\right)\right|>\delta . \end{array}\right. \end{array}$$

The estimation model based on Long and short-term memory network can be divided into three types: average loss function, absolute loss function, and classification loss function. In order to better analyze the variation relationship between the three loss methods and corresponding data, the loss function and corresponding curve are obtained, as shown in Figure 10. It can be seen from Figure 10 that the curves corresponding to several different loss functions have typical symmetry characteristics. It can be seen from the test data that with the increase of *x*, the corresponding loss of the curve first slowly decreases to the lowest point and then gradually increases. The average loss curve absolute loss curve and classified loss curve also showed a relatively obvious trend of decreasing first and then increasing. It can be seen from the absolute value loss function and classification loss function that its linear characteristics are relatively obvious. When *x* value is constant, the data corresponding to the average loss amount is the largest, while the loss amount corresponding to the absolute loss function and the classified damage function is basically the same.

## 4. Feasibility Study on Psychological Rehabilitation Training of Volleyball Players Based on Artificial Intelligence Calculation

### 4.1. Feasibility Analysis of Psychological Health Training Methods for Volleyball Players

Volleyball players' mental health and corresponding training methods are very complex, and corresponding mental health and training methods are very important for volleyball players. A good mental health mood can improve the training level and skills of volleyball players. In order to further analyze the emotional changes of volleyball players in the process of mental health training, five different evaluation indexes are obtained through summary analysis: *A*-Motor skills; *B*-Mental training, *C*-Verbal cues, *D*-Mood regulation, *E*-Health training. These five indicators can reflect the training methods and feasibility analysis of volleyball players' mental health from different aspects. Different indicators can be used for quantitative analysis of the model.

In order to further study the proportion of five different indicators in volleyball players' mental health training, the proportion of volleyball players' mental health under the effect of different indicators was obtained through summary analysis, as shown in Figure 11. According to the proportion analysis in the figure, it can be seen that motor skills account for the smallest proportion, only 5%, while psychological training and mood regulation account for the same proportion, both 25%. Verbal cues accounted for the most, about 35 percent, and health training accounted for about 10 percent.

### 4.2. Research on Artificial Intelligence Technology in Volleyball Players' Mental Health Training Methods

By combining the Kalman filter algorithm mentioned above, and by derivation and parameter estimation of neural network algorithm and long and short-term memory network algorithm, the corresponding model of volleyball players' mental health training method under the effect of artificial intelligence can be obtained, and the corresponding estimation test can be carried out [35, 36]. In order to further quantitatively analyze the psychological health training indicators of volleyball players under the effect of artificial intelligence, a mental health training flow chart with artificial intelligence technology was obtained through comparative analysis, as shown in Figure 12. It can be seen from the process in the figure that: first, the model data is imported into the data initialization module, and the corresponding targeted indicators are obtained through the initial analysis of the data. Then the targeted indexes are imported into the data preprocessing module. The data is then imported into the training and verification modules and calculated by building a two-way LSTM network. The calculated data will be introduced into the training plate of the model and judged by the evaluation indicators. If it meets the requirements, it will be imported into the training method for feasibility study. If it does not meet the requirements, it will be imported into the parameter adjustment for parameter optimization, and continue to carry out iterative analysis.

Through the above description, the corresponding calculation process of mental health training method based on artificial intelligence technology can be obtained. Firstly, the Kalman filter algorithm and neural network algorithm in the artificial intelligence model are analyzed, and then the long and short-term memory network is evaluated. Then artificial intelligence calculation is used to estimate and analyze the relevant models, and finally, the corresponding optimization model is obtained. Model data are imported into the optimization model, and corresponding calculation results of mental health training can be obtained through calculation, as shown in Figure 13. As can be seen from the three-dimensional bar chart in the figure, the curve of the first evaluation parameter shows a trend of gradual decline with the gradual increase of the index. The second evaluation parameter shows a trend of gradual increase, and conforms to the rule of linear change, corresponding to a relatively large range of change. With the increase of the third evaluation parameter, the corresponding data still shows a trend of gradual increase, but the range and amplitude of change are relatively small. The data corresponding to the evaluation parameters in Chapter 4 has obvious fluctuation characteristics, while the variation range and range of the fifth evaluation parameter are relatively small.

## 5. Discussion

The artificial intelligence model is used to estimate the neural network and long and short-term memory network, so as to obtain the corresponding calculation model. The model is used to analyze and evaluate different indicators. In order to further analyze the accuracy of the model, the model is verified by comparing test data with model data. The corresponding comparison curve of mental health training was obtained through calculation and comparison, as shown in Figure 14. According to the proportion of the two kinds of data in the figure, it can be seen that the model data is basically consistent with the experimental data, which indicates that the optimization model can better reflect the accuracy of the corresponding indicators of the actual training method. Volleyball players' mental health training is very important. We can use mental health, mood adjustment, sports skills optimization, and other ways to analyze the feasibility of sports methods, so as to get the latest optimization results.

## 6. Conclusion

1. In the parameter variation curve, the variation range of weight is the smallest, indicating that its influence on the output value is relatively small. The variation trend of the function increases first and then decreases, and its influence on the output value decreases gradually. The data corresponding to the threshold shows an obvious fluctuation trend on the whole, and the fluctuation range is relatively large, indicating that it has the greatest influence on the output result.
2. The error curves under different evaluation indexes show obvious fluctuation characteristics, and the linear and non-linear characteristics of the curves are obvious. The corresponding data increase first and then decrease, and the corresponding increase stage conforms to linear change. Four different evaluation indexes can better reflect the changing rules of actual model data.
3. The data can be normalized by using artificial intelligence technology. Through calculation, it can be seen that the maximum curve first drops to the lowest point and then slowly rises. The corresponding minimum value changes steadily at first, then increases rapidly under data mutation, and finally increases the maximum value gradually.

## Figures and Tables

**Figure 1:** Flow chart of artificial intelligence algorithm.

**Figure 2:** Time update curve.

**Figure 3:** Status update curve.

**Figure 4:** Neural network calculation process and learning method.

**Figure 5:** Parametric curve.

**Figure 6:** Activation function.

**Figure 7:** Long and short-term memory network output.

**Figure 8:** Appraisal curve.

**Figure 9:** Normalized curve.

**Figure 10:** The curve corresponding to the loss function.

**Figure 11:** Health training indicators.

**Figure 12:** Mental health training flow chart based on artificial intelligence calculation.

**Figure 13:** Mental health training results based on artificial intelligence calculation.

**Figure 14:** Contrast curve of mental health training.

## Data Availability

The datasets used during the current study are available from the corresponding author on reasonable request.
